# MRI Imaging Omics and Risk Factors Analysis of PWMD in Premature Infants Based on Fuzzy Clustering Algorithm

This article has been retracted.

**DOI:** 10.1155/2022/8624617

**Published:** 2022-09-29

**Authors:** Xiaofei Wang, Yuewen Hao, Huan Sun, Chao Chen

**Affiliations:** ^1^Department of Radiology, Xi'an Children's Hospital, Xi'an 710003, China; ^2^NICU, Xi'an Children's Hospital, Xi'an 710003, China

## Abstract

The magnetic resonance imaging (MRI) characteristics of periventricular white matter damage (PWMD) in premature infants using the fuzzy c-means clustering algorithm (FCM) is explored, and the influencing factors are further clarified. A total of 100 premature infants admitted to the neonatal department of our hospital from February 2020 to February 2022 are selected for in-depth investigation. According to the occurrence of PWMD, they are divided into the PWMD group and the simple premature delivery group, with 50 cases in each group. All preterm infants are examined by MRI and the changes in image characteristics and apparent diffusion coefficient (ADC) values are analyzed. Clinical information of the subjects is collected and the influencing factors of PWMD in preterm infants are analyzed by multivariate regression analysis. In the first magnetic resonance imaging (MRI) examination, the cases of punctured, clustered, and linear lesions are 28 cases, 12 cases, and 10 cases, respectively. The experimental results showed that PWMD of preterm infants presented punctate, clustered, and high linear T1 signal MRI manifestations, which caused a downward trend of ADC value, and caused respiratory distress, low birth weight, premature rupture of membranes, respiratory tract infection, and other risk symptoms.

## 1. Introduction

White matter is a nerve fiber that controls the shared signals of neurons and is mainly aggregated and synthesized by axon aggregates of most neurons, playing an important coordinating role in the normal operation of brain regions [1, 2]. Premature infants have immature cerebrovascular development, and their oligodendrocytes are highly sensitive to inflammatory response and tissue hypoxia, resulting in cerebral white matter damage in premature infants, of which the most common one is periventricular white matter damage (PWMD), accounting for more than 80.00%. In severe cases, ventricular voice-over transformation will occur, which will increase the incidence of neurological sequelae such as cerebral palsy, cognitive impairment, and audio-visual dysfunction in premature infants, and the risk of sequelae will be affected by birth weight, gestational age, and other factors and will change accordingly [3]. Magnetic resonance imaging (MRI) is a commonly used technology in clinical imaging examination, which is widely used in the diagnosis of many diseases and has been unanimously recognized by experts. Fuzzy C-means clustering algorithm (FCM) assisted MRI brain image segmentation has achieved certain results in the field of medical and computer image processing [4, 5].

At present, there is no unified view on the clinical mechanism, pathological changes, and magnetic resonance imaging changes of PWMD injury, and it has become a hot research direction at home and abroad. Therefore, quantitative analysis of the clinical mechanism, imaging characteristics, and influencing factors of premature PWMD has important guiding significance for later prevention and treatment. The purpose of this study is to analyze the MRI influence characteristics of premature infants with PWMD assisted by FCM technology, and to further analyze the influencing factors of premature infants with PWMD, so as to provide data support for the subsequent diagnosis, prevention, and treatment of premature infants with PWMD.

The rest of this paper is organized as follows: Section 2 discusses the related work, followed by clinical case information and treatment plan designed in Section 3.  Section 4 shows the experimental results, and Section 5 summarizes the full-text primary coverage and points to future research directions.

## 2. Related Work

FCM algorithm can make the use of iterative optimization objective function for the fuzzy partition of a data set, the application of the technology of MRI image such as image segmentation can effectively solve the problem of threshold setting and multiple branch division. It has high applicability in the characteristics of image uncertainty and fuzziness, at the same time, this algorithm does not need human intervention to supervise. Image segmentation can be automatically completed. In this study, the FCM algorithm was used to assist in MRI image examination of premature infants, which can obtain image results with high segmentation accuracy and provide a basis for MRI image diagnosis [6]. Clinical premature occurrence PWMD diagnosis depends on imaging technology, more commonly used, including ultrasound, CT, and MRI, CT detection has great radiation dose and diagnostic sensitivity and specificity is lower than the diagnostic criteria, ultrasonography can only be a sensitive and effective diagnosis of the cystic lesion, sensitivity in the diagnosis of children with cystic lesion is poorer. MRI technology has high image resolution and can clearly display the boundaries of gray matter and white matter, just to provide a more accurate and reliable image basis [7]. Yang et al. [8] believed that the main MRI manifestations of PWMD in premature infants were point-like, cluster-like, and line-like T1 strong signal and point-like damage was easily absorbed. According to the results of this study, PWMD routine MRI examination results are dotted, tufted, and high linear T1 signal performance, with or without low T2 signal. It can be seen that most of the spots and clusters of lesions disappeared, and a few cases further developed into periventricular leukomalacia (PVL). This result is consistent with the above literature, and the risk of PVL development is higher in linear lesions. The reason may be that punctured and clustered lesions are easy to be absorbed and gradually absorbed over time, while the lesion area of linear lesions is large and difficult to be absorbed, which leads to further expansion and formation of the cystic lumen and the eventual development of PVL [9]. Combined with the apparent diffusion coefficient (ADC) value analysis of this study, the ADC value of the PWMD group was significantly lower. The reason for this result is that diffusion-weighted imaging technology can reflect the irregular movement of water molecules in tissues. The change in water molecules' movement will directly affect the signal strength, and the ADC value can be calculated according to the change in signal strength. Therefore, the ADC value can be used as a sensitive indicator of signal intensity. Na^+^-K^+^ -ATPASE on the membrane of children in the early stage of ischemia is dysfunctional, which leads to cytotoxic brain edema, and ultimately inhibits the diffusion movement of water molecules in cells, resulting in reduced ADC value and the high signal performance of DWI [10].

Studies have shown that birth weight and gestational age are factors affecting the incidence of PWMD in premature infants [11]. The results were consistent with the results of this study, which showed that respiratory distress, low birth weight, premature rupture of membranes, and respiratory tract infection were risk factors for PWMD in premature infants.

The reason why respiratory distress increases the risk of PWMD may be that immature pulmonary surfactant causes pulmonary ventilation dysfunction, which prevents premature infants from obtaining sufficient oxygen through ventilation, and carbon dioxide in the body cannot be discharged from the body normally through ventilation, resulting in the destruction of acid-base balance in premature infants, which in turn lead to brain tissue hypoxia and proinflammatory factor, oxygen-free radical release in great quantities. This makes children's brain in a passive pressure flow state, the body's ability to regulate the response is impaired, under the stimulation of oxygen and inflammation, immature oligodendrocyte axons swelling necrosis, leading to brain white matter lesions [12].

Incandescent water sensitivity and cerebral vascular regulation in low birth weight preterm infants: oligodendrocytes, oxygen sensitivity, and immune system function development are not yet mature, in the face of environmental stimuli such as hypoxia and ischemia, and inflammation can be collected by the regulation system of specific interventions to improve, in anaerobic infection, under the influence of factors such as damage to deep brain white matter, and stimulates release of oxygen-free radicals and proinflammatory factor. It increases the permeability of white matter medullary vein in brain tissue and causes current lesions [13].

Infection is the main reason for the natural preterm birth and intrauterine infection can cause premature rupture of membranes, mother pregnancy infection after a large number of the secretion of inflammatory medium to further activate the heat production center. This causes fever, which indirectly causes the fetus to consume more oxygen and increase its body temperature, leading to oxygen supply to the fetus's brain cells and causing brain damage. Additional infection during pregnancy can make interleukin and tumor necrosis factor and inflammatory medium, vasculitis, and cytokines lead to pregnant women and fetus hematic disease, fetal brain tissue oligodendrocytes and radial glial cells produced in great quantities, and the above two types of cell excessive proliferation can cause brain damage, serious can form cerebral palsy [14].

A respiratory infection can inhibit lung surface after the synthesis and secretion of active substance and reduce its efficiency, in children with prolonged breathing difficulties, indirect degree increased breathing difficulties caused by the shortage problem of oxygen intake, causing huge accumulation of acid chemicals in the body at the same time, combined with the inflammation, thus hindering the myelin formation, resulting in brain injury [15].

This research is still insufficient smaller sample size and variable selection is not comprehensive, may affect the overall research to the conclusion. Follow-up studies can screen out more PWMD-related clinical cases for analysis and can also be studied and discussed from different perspectives of MRI and other imaging techniques in the diagnosis of preterm infants.

## 3. Clinical Case Information and Treatment Plan

### 3.1. Clinical Case Information

A total of 100 premature infants admitted to the department of neonatology of our hospital from February 2020 to February 2022 are selected for the study. According to the occurrence of PWMD, they are divided into the PWMD group and the simple preterm birth group, with 50 cases in each group. Gestational age ranged from 30 to 36 weeks, with an average of (34.21 ± 1.12) weeks. Body weight ranged from 1500 to 2500 g, with an average of (1360.34 ± 132.12) g. Inclusion criteria: preterm production, it can tolerate MRI examination; the children's family members clearly defined the study content and voluntarily signed the consent form. Exclusion criteria: chromosomal abnormalities, neurodevelopmental malformation, and brain damage caused by hereditary metabolic disorders; Incomplete clinical information; Contraindications of MRI examination; and an infectious disease.

### 3.2. Treatment Plan

MRI scanning scheme: GE Discovery MR 750 3.0 Tesla scanner (GE Medical System, WI, USA) is used for MRI scanning and data collection of the subjects. The 32-channel head coil is used to receive MRI signals. The subjects are supine and their heads are filled with sponge foam pads. Then, conventional MRI scanning is performed, including T1WI and T2WI scanning. The TR parameter of T1WI scanning is 640 ms, the TE parameter is 10 ms, the FOV parameter is 22 cm × 22 cm, the matrix parameter is 288 × 192, the NEX parameter is 1, the layer thickness parameter is 4.5 mm, and the layer spacing parameter is 4 mm. TR, TE, FOV, matrix, NEX, layer thickness, and layer spacing parameters are 3936 ms, 85 ms, 22 cm × 22 cm, 288 × 244, 2, 4.5 mm, and 4 mm, respectively. A gradient magnetic field is applied from the *X*, *Y,* and *Z* axes. The parameters of B value are set as 0 s/mm and 1000 s/mm. The parameters of TR, TE, FOV, and matrix are set as 2123 ms, 56 ms, 22 cm × 22 cm, and 160 × 160 for DWI scanning. NEX parameter is 4, layer thickness parameter is 4.5 mm, and layer spacing parameter is 4 mm. The DWI is recorded into GE AW4.6 workstation Functool software and converted into AN ADC map to measure the ADC value of the region of interest.

FCM calculation method is as follows: the FCM algorithm is used to assist the analysis of MRI image segmentation, and the fuzzy weight index *M*, classification number *C*, and *ε* parameters are set to 2, 4, and 0.001 and then calculated.

### 3.3. Statistical Methods

All statistical analyses are performed by SPSS 24.0 statistical analysis software. The measurement data are described by mean ± standard deviation $\left(\bar{x}\pm s\right)$, and the *T* test is used. The counting data are described by the number of cases and composition ratio [*n*, (%)], and the Chi-square test is used. Multivariate logistic regression analysis of the influencing factors of premature infants with PWMD: *P* < 0.05, the difference is statistically significant.

## 4. Experimental Results

### 4.1. Changes of MRI Characteristics in the PWMD Group

The first MRI examination shows that 28 cases have punctured lesions with a diameter <5 mm and the number of lesions is less than 3, presenting a distributed distribution, 12 cases are clustered lesions and 10 cases are linear lesions, with the number of lesions ranging from 4 to 10.  Figure 1 shows the initial examination of punctured PWMD MRI.  Figure 2 shows the cluster PWM DMRI for the first time.  Figure 3 shows the first examination of linear PWMD MRI. Through the above experimental results, it can be observed that there are 8 cases with a strong signal on DWI and normal MRI, 31 cases with a strong signal on DWI and strong signal on MRI, with or without a low signal on T2, and 12 cases with normal DWI and strong signal on MRI, with or without low signal on T2.  Figure 4 shows the point-shaped PWMD MRI review.  Figure 5 shows the cluster PWM DMRI review.  Figure 6 shows the linear PWMD MRI review. Through the above experimental results, it can be observed that the lesions disappeared completely in 28 premature infants with point injury, 8 of the 12 cases with cluster injury disappeared completely, 4 of the 12 cases developed PVL, and 4 of the 10 cases with linear injury developed PVL, and 6 of the lesions disappeared completely.

### 4.2. Differences in MRI ADC Values between the PWMD Group and the Simple Preterm Birth Group

Both Table 1 and Figure 7 show the differences in ADC values in MRI examination. It can be seen clearly from Table 1 and Figure 7 that the PWMD group have significantly lower ADC values in the focal area than the preterm preterm group (*P* < 0.05).

### 4.3. Univariate Analysis of Differences in Clinical Data of PWMD

Table 2 shows the univariate analysis of differences in clinical data of PWMD. It can be seen from Table 2 that the proportions of respiratory distress, low birth weight, premature rupture of membranes, and respiratory tract infection are higher in PWMD group and the differences are statistically significant (*P* < 0.05).

### 4.4. Influencing Factors of PWMD in Premature Infants

Table 3 is the variable assignment table.  Table 4 shows the analysis of influencing factors of PWMD in premature infants by logistic regression. It is clearly evident from Table 3 and Table 4 that respiratory distress, low birth weight, premature rupture of membranes and respiratory tract infection are all risk factors for PWMD in premature infants (*P* < 0.05).

## 5. Conclusion

This study analyzes the MRI influence characteristics of premature infants with PWMD assisted by FCM technology. MRI of premature infants with PWMD shows point-like, cluster-like, and linear T1 hyperintensity, with or without T2 hyperintensity, and ADC value would be significantly reduced. Premature infants with respiratory distress, low birth weight, premature rupture of membranes, respiratory tract infection, and other risk factors for premature PWMD should be diagnosed by MRI in a timely manner.

## Figures and Tables

**Figure 1:** Initial examination of punctured PWMD MRI.

**Figure 2:** Cluster PWMD MRI for the first time.

**Figure 3:** First examination of linear PWMD MRI.

**Figure 4:** Point-shaped PWMD MRI review.

**Figure 5:** Cluster PWMD MRI review.

**Figure 6:** Linear PWMD MRI review.

**Figure 7:** Differences of ADC values in MRI examination.

**Table 1:** Differences of ADC values in MRI examination.

Group	ADC
PWMD group	942.12 ± 168.67
Simple preterm delivery group	1531.23 ± 109.43
*T*	−20.719
*P*	<0.001

**Table 2:** Univariate analysis of differences in clinical data of PWMD.

Metric	PWMD group	Simple preterm delivery group	*t*/*x*^*2*^	*P*
Gestational age	34.21 ± 1.12	34.18 ± 1.09	0.071	0.943

Sex			0.378	0.539
Man	32 (64.00)	29 (58.00)		
Woman	18 (36.00)	21 (42.00)		

Respiratory infection			6.112	0.013
Yes	37 (74.00)	25 (50.00)		
Deny	13 (26.00)	25 (50.00)		

Premature rupture of fetal membranes			6.986	0.008
Yes	36 (72.00)	23 (46.00)		
Deny	14 (28.00)	27 (54.00)		

Respiratory distress			5.769	0.016
Yes	32 (64.00)	20 (40.00)		
Deny	18 (36.00)	30 (60.00)		

LBW			4.889	0.027
Yes	33 (66.00)	22 (44.00)		
Deny	17 (34.00)	28 (56.00)		

**Table 3:** Variable assignment table.

Metric	Variable	Assignment
Respiratory infection	*X*1	1 = yes, and 2 = No
Premature rupture of fetal membranes	*X*2	1 = yes, and 2 = No
Respiratory distress	*X*3	1 = yes, and 2 = No
LBW	*X*4	1 = yes, and 2 = No
PWMD	*Y*	1 = yes, and 2 = No

**Table 4:** Analysis of influencing factors of PWMD in premature infants by logistic regression.

Influencing factor	*B*	S.E.	Wald	*P*	OR	95% CI
Respiratory infection	2.134	0.990	4.645	0.031	8.445	1.213 ∼ 58.788
Premature rupture of fetal membranes	8.281	2.224	13.862	<0.001	94.861	50.491 ∼ 308.708
Respiratory distress	2.948	1.306	5.100	0.018	3.074	1.476 ∼ 16.444
LBW	2.251	0.835	7.205	0.007	9.511	1.836 ∼ 49.264

## Data Availability

The simulation experiment data used to support the findings of this study are available from the corresponding author upon request.
